The article "Effects of Gemcitabine and Oxaliplatin Combined with Apatinib on Immune Function and Levels of SIL-2R and sicAM-1 in Patients with Gallbladder Cancer" was retracted in 2023. Reasons: signs of a paper mill; suspected computer-generated content; unreliable results or conclusions; concerns about the data.

# Effects of Gemcitabine and Oxaliplatin Combined with Apatinib on Immune Function and Levels of SIL-2R and sicAM-1 in Patients with Gallbladder Cancer

**DOI:** 10.1155/2022/4959840

**Published:** 2022-08-25

**Authors:** Linlin Qu, Kun Li, Kui Liu, Weiyu Hu

**Affiliations:** Department of Hepatopancreatobiliary Surgery, The Affiliated Hospital of Qingdao University, Qingdao 266000, China

## Abstract

**Objective:**

The aim of this study was to determine how gemcitabine, oxaliplatin combination, and apatinib affect immune function and SIL-2R and sicAM-1 levels in patients with gallbladder cancer.

**Methods:**

Retrospective analysis of 116 patients with gallbladder cancer treated at our institution between February 2019 and February 2021. The patients were randomly divided into control and study groups, with 58 patients in each group. The study group received the combination of apatinib and the control group received gemcitabine and oxaliplatin. Immune function, serum tumor markers, short-term efficacy, survival measures, and incidence of adverse events were monitored and compared between the two groups.

**Results:**

CD3+, CD4+, CD4+/CD8+, and NK levels were significantly higher in both groups after treatment, while CD8+ levels were significantly lower; levels of sicAM-1, sicAM-1 (VEGF), and CEA were greatly reduced in both groups after treatment; there were significant differences between the study and control groups in terms of rr46.55% and DCR84.48%; at one year after treatment, the survival rate in the study group increased from 67.24% in the control group to 79.31%, with an increase in both PFs and 0S. Compared with the control group, the incidence of hypertension and myelosuppression, neutropenia, proteinuria, and hand-foot syndrome were lower in the study group (*P* < 0.05). All differences were statistically significant.

**Conclusion:**

In the treatment of gallbladder cancer, the use of gemcitabine and oxaliplatin combined with apatinib can effectively control the progression of patients' disease.

## 1. Introduction

Gallbladder cancer is a relatively common malignant tumor of the biliary system in clinical practice, with insidious onset, rapid tumor growth, and high malignancy, which is a great threat to patients' lives [1]. The occurrence of gallbladder cancer is related to various risk factors, such as gallbladder stones, bile duct inflammation, and obesity, but the exact etiology is still unclear [2, 3]. In the process of continuous in-depth clinical research on gallbladder cancer, the treatment methods about gallbladder cancer have been continuously improved, and the treatment effect of gallbladder cancer has been significantly enhanced [4, 5]. Due to the high malignancy of gallbladder cancer, chemotherapy can directly kill tumor cells [6, 7]. Gemcitabine, oxaliplatin, and apatinib all have significant effects on the treatment of tumors [8, 9]. Gemcitabine has a strong broad-spectrum antitumor activity and a unique mechanism of action and is widely used in the treatment of malignant tumors in clinical practice; oxaliplatin has the advantage of significant effects and few adverse effects; and apatinib is able to antagonize vascular endothelial growth factor receptor 2 (VEGFR-2) and can effectively promote apoptosis of tumor cells. In this paper, the efficacy of gemcitabine and oxaliplatin combined with apatinib in the treatment of gallbladder cancer is analyzed and reported as follows.

The article "Effects of Gemcitabine and Oxaliplatin Combined with Apatinib on Immune Function and Levels of SIL-2R and sicAM-1 in Patients with Gallbladder Cancer" was retracted in 2023. Reasons: signs of a paper mill; suspected computer-generated content; unreliable results or conclusions; concerns about the data.

## 2. Material and Methods

### 2.1. General Material

Patients with gallbladder cancer admitted to our hospital between February 2019 and January 2021 were randomly divided into two groups: 23 males and 35 females in the control group, aged 42–76 years; 58 patients in the study group, with a mean age of 56.08 years and a mean disease duration of 15.09 months (see Table 1), with a performance status (ECOG) score of 1 in 11 cases, 2 in 20 cases, 3 in 27 cases, and tumor patients 1 case with score 4 and TNM stage [10] (tumor node metastasis grading). A total of 17 cases of stage III and 41 cases of stage IV were found; in the study group, there were 24 males and 34 females, with ages ranging from 41 to 77 years, mean age (57.12 ± 4.25) years, and duration of disease (15.12 ± 2.01) months. Scores of ECOG: 12 cases were 1, 20 cases were 2, and 26 cases were 3. 15 cases were classified as stage III according to TNM, and 43 cases were stage IV. The differences between the two groups in terms of gender, age, and disease duration were not statistically significant. The control group was given gemcitabine and oxaliplatin, while the experimental group added apatinib to the control group. The medical ethics committee of the hospital has approved the study.

### 2.2. Criteria of Inclusion and Exclusion

Inclusion criteria were ① Compliance with the guidelines of the Biliary Surgery Group of the Chinese Medical Association for the diagnosis of gallbladder cancer [11]; ② confirmed by cell immunology, imaging examination, and pathological biopsy of gallbladder cancer; ③ aged 18–80 years old, with the first gallbladder cancer; ④ ECOG score of 1–3; TNM stage of stage III–IV; ⑤ estimated survival time >3 months, which could not be treated by previous surgery or drugs; ⑥ have the solid lesions that can be measured (the diameter of the lesions in the spiral CT examination is ≥10 mm); ⑦ patients and members of their families get an explanation of the study's goals, and they sign an informed consent form as a proof of their agreement.

The article "Effects of Gemcitabine and Oxaliplatin Combined with Apatinib on Immune Function and Levels of SIL-2R and sicAM-1 in Patients with Gallbladder Cancer" was retracted in 2023. Reasons: signs of a paper mill; suspected computer-generated content; unreliable results or conclusions; concerns about the data.

Exclusion criteria were ① Patients with injury or dysfunction of heart and blood vessels and other organs; ② patients with obvious gastrointestinal bleeding, including local ulcer, hematochezia and hematemesis within two months, and patients with occult blood in stool; ③ patients with primary gastric cancer without surgical resection, who are often considered to have massive gastrointestinal bleeding without examination; ④ there are no other diseases of the gallbladder, such as gangrenous cholecystitis, gallbladder atrophy, and diffuse stones; ⑤ abnormal coagulation function, allergic to research drugs; ⑥ accompanied by cognitive impairment and mental disorders; ⑦ poor compliance, recently participated in other clinical drug researchers.

### 2.3. Research Methods

After admission, the patients underwent relevant examinations, including laboratory, cytology, imaging, and pathological examination, and were given basic treatment, including analgesia, sedation, anti-inflammatory, anti-infection, and nutritional support. Gemcitabine and oxaliplatin were used in the control group: 1000mg/m2 gemcitabine (Jiangsu Hausen Pharmaceutical Group Co. Ltd. Chinese medicine standard word H20030104) was dissolved in 100 ml of 0.9% normal saline for 30 minutes, once/week, 3 weeks/course, and then entered a course after one week's rest; 85 mg/m^2^ oxaliabine Fireseuskaby (Wuhan) Pharmaceutical Co. intravenous instillation for 2.5∼3 hours, 2 weeks/time, 2 weeks/course of treatment, one week of intermediate rest, and then enter a course of treatment for 4 months. Following this, apatinib, a drug manufactured by Jiangsu Hengrui Pharmaceutical Co. Ltd. and given in warm water, 500 mg/time, once a day, 30 minutes after meals, and for two courses of treatment was administered to the research group. Testing for gastrointestinal, liver, and kidney functions should be done as soon as possible if side effects such as nausea and vomiting occur during chemotherapy. If the white blood cell level is abnormally increased, the electrocardiogram, liver, and kidney function shall be monitored regularly; if the white blood cell level is abnormally decreased, the granulocyte colony stimulating factor treatment shall be implemented; and if bone marrow suppression occurs, the hematopoietic factor shall be injected.

### 2.4. Observational Indicators

① Immune function measurement: Flow cytometry (Nexcelom Bioscience Company, USA) identified T cell subsets, in peripheral venous blood before and 2 months after the natural killer cell. ② Evaluation of sICAM-1, vascular endothelial growth factor, and carcinoembryonic antigen before and after therapy was conducted. A nocturnal blood sample was taken from the patient and then centrifuged in the morning. For cold storage, the supernatant was gathered. In this research, flow cytometry was used to measure sIL-2R and sICAM-1 levels. Shanghai BRahman State Biotechnology Co. Ltd. provided the kit, and the double antibody Sandwich method was used to measure VEGF and CEA levels. Operate in line with the instructions provided in the package.③ Clinical treatment effect: complete response (CR): complete tissue disappeared completely without tumor enhancement >4 weeks; partial response (PR): a reduction in lesion tissue of at least 50% and a duration of at least four weeks are required; stable disease (SD): lesions on the largest scale dropped by 50% or rose by 25%, but no new lesions formed; progressive disease (PD): lesion tissue grew by more than 25%, or a new lesion was discovered. Disease control rate (DCR) = (CR + PR + SD) cases/total cases *x* 100%; objective response rate (RR) = (CR + PR) cases/total cases 100%. ④ Survival indicators: follow-up (outpatient, SMS, telephone, etc.) and record the survival indicators of the two groups during one year, including survival rate, survival time, progression-free survival (progression-free survival,PFs), and overall survival (0 s). Survival was the cumulative survival ratio after the first year of follow-up. The PFs and 0 s reflect the amount of time elapsed between the time of enrollment and the time of death or the last follow-up, respectively. ⑤ Adverse reactions: patients experienced hypertension, neutropenia, and proteinuria as well as bone marrow suppression and hand-foot syndrome throughout therapy and follow-up.

The article "Effects of Gemcitabine and Oxaliplatin Combined with Apatinib on Immune Function and Levels of SIL-2R and sicAM-1 in Patients with Gallbladder Cancer" was retracted in 2023. Reasons: signs of a paper mill; suspected computer-generated content; unreliable results or conclusions; concerns about the data.

### 2.5. Statistical Treatment

Using SPSS 24.0 statistical software, *t*-tests were employed to compare groups, and measurement data according to a normal distribution was presented as ±. For comparisons between groups, enumeration data were reported in terms of number of cases and percentages (*n* and %), and a *P* < 0.05 denotes statistically significant differences.

## 3. Outcome

### 3.1. Comparison of Immune Function

Immunological parameters were not significantly different before treatment. There was a striking increase in CD3+, CD4+, CD4+/CD8+, and NK in NK cells and a striking decrease in CD8+ in NK cells. CD3+, CD4+/CD8, and NK levels in the study group were significantly higher than CD4+/CD8+ levels in the control group; see Table 1 and Figure 1.

### 3.2. Comparison of Serum Tumor Markers

In the comparison of serum tumor markers, the levels of sIL-2R, sICAM-1, VEGF, and CEA were flatly lower in the control group than in the study group as shown in Table 2 and Figure 2.

The article "Effects of Gemcitabine and Oxaliplatin Combined with Apatinib on Immune Function and Levels of SIL-2R and sicAM-1 in Patients with Gallbladder Cancer" was retracted in 2023. Reasons: signs of a paper mill; suspected computer-generated content; unreliable results or conclusions; concerns about the data.

### 3.3. Comparison of Clinical Therapeutic Effects

In terms of clinical efficacy, the RR after treatment was 46.55% higher and the DCR was 84.48% higher in the study group than in the control group, and the differences were statistically significant as shown in Table 3 and Figure 3.

### 3.4. Comparison of Survival Indicators

In the comparison of survival indicators, the one year survival rate after treatment was 79.31% higher in the study group than in the control group (*P* < 67.24%), which is remarkable.  Table 4 and Figure 4 show that the survival time, PFs, and 0 s were longer in the study group than in the control group.

### 3.5. Comparison of Adverse Reaction Rates

In the comparison of the incidence of adverse reactions, hypertension and myelosuppression were lower in the study group, but the differences were not statistically significant. Neutropenia, proteinuria, and hand-foot syndrome were quite rare in the study group as shown in Table 5 and Figure 5.

## 4. Discussion

The main treatment modality for malignant tumors is comprehensive treatment, and radical resection is the only way to treat patients with gallbladder cancer with the possibility of cure [12]. Patients with gallbladder cancer need to undergo surgical exploration first, and resection at an early stage can effectively prolong the survival time of patients [13]. However, in actual clinical practice, many patients with gallbladder cancer are diagnosed in the middle and late stages because of the early manifestations of the disease and the rapid growth of the tumor, and the tumor cells have already invaded the plasma membrane, resulting in metastases in the liver and peritoneum [14]. Patients with advanced gallbladder cancer have long operation time, large resection area, high surgical risk, and many postoperative complications [15]. Therefore, chemotherapy has become the main treatment modality for this group of patients. Among them, gemcitabine, oxaliplatin, and apatinib as chemotherapy drugs have different anticancer effects and mechanisms, which can amazingly promote apoptosis of diseased tissues to inhibit the growth and metabolism of tumor cells [16]. Currently, the anticancer mechanisms and effects of gemcitabine, oxaliplatin, and apatinib are frequently studied at home and abroad, while the effects of gemcitabine, oxaliplatin, and apatinib on immune function, sIL-2R, and sICAM-1 are still relatively limited [17]. In this study, gemcitabine and oxaliplatin combined with apatinib significantly inhibited tumor vascular growth, improved somatic cell immune function, alleviated sIL-2R, and sICAM-1 levels, improved short-term treatment effects and survival time, and controlled the occurrence of adverse effects.

The article "Effects of Gemcitabine and Oxaliplatin Combined with Apatinib on Immune Function and Levels of SIL-2R and sicAM-1 in Patients with Gallbladder Cancer" was retracted in 2023. Reasons: signs of a paper mill; suspected computer-generated content; unreliable results or conclusions; concerns about the data.

When cancer cells invade the gallbladder, immune function is suppressed, allowing the growth and development of tumor vascular cells, and increasing the activity of tumor biomarkers. This leads to a dramatic decrease in CD3 +, CD4 +, CD4 +/CD8 +, and NK levels, an increase in CD8 + and a decrease in anticancer and anti-infective capacity. The literature[18] treats breast cancer patients with gemcitabine, which interferes with the expression of VEGF and its receptor in cancer cells by engaging the AKT pathway, thereby promoting apoptosis of tumor cells. Consistent with previous studies, gemcitabine, oxaliplatin, and apatinib have been shown to improve immune function, inhibit tumor cell activity, and reduce the activity and expression of serum tumor markers in patients with gallbladder cancer [19]. As a nucleoside analogue, gemcitabine can effectively affect DNA synthesis during tumor cell metabolism and induce apoptosis in cancer cells. Oxaliplatin, a third-generation anticancer drug, has similar effects to gemcitabine and is involved in the growth and proliferation of tumor cell DNA. Apatinib, as a VEGFR-2 tyrosine kinase inhibitor, can effectively bind to the VEGF receptor, inhibit its expression in tumor cells, and interfere with the growth, metabolism, and proliferation of tumor blood vessels. It can also regulate the activity of tumor markers, such as sIL-2R and sICAM-1, whose synergistic effects can alleviate cancer cell-induced immune disorders, promote body immune regulation, improve immune function, and enhance therapeutic efficacy.

Chemotherapy and targeted drugs are often used to treat patients with biliary tract cancer. Among them, chemotherapeutic drugs have a strong suppressive effect on the body's immune system and are prone to adverse reactions and drug resistance, which affect prognosis and safety. In recent years, there has been an explosion of research on targeted drugs. The positive effects of cancer treatment have become more pronounced and the side effects have been greatly reduced. The literature [20] demonstrated that oxaliplatin and apatinib, adjuvant therapy for patients with locally advanced biliary tract cancer can significantly improve DCR and therapeutic benefits and enhance anticancer activity. Apatinib was safe and effective, and no deaths were reported. The literature [21] showed that gemcitabine, oxaliplatin, and apatinib significantly improved the short- and long-term outcomes and reduced the incidence of adverse effects in patients with biliary cancer. This finding is consistent with a previous study by [22] et al. Improved treatment outcomes and increased overall survival time have been shown in patients with gallbladder cancer in a manner that is both very safe and within the tolerable range of possible side effects [23].

The article "Effects of Gemcitabine and Oxaliplatin Combined with Apatinib on Immune Function and Levels of SIL-2R and sicAM-1 in Patients with Gallbladder Cancer" was retracted in 2023. Reasons: signs of a paper mill; suspected computer-generated content; unreliable results or conclusions; concerns about the data.

There are certain limitations in this study, mainly including limited sample size, deviation of the study results from actual clinical data, which affects the reliability of the study report; insufficient time to assess the long-term effectiveness and resistance to treatment; and failure to consider the effects of drug treatment on other immune mechanisms. Expanding the sample size, extending the follow-up period, and studying different mechanisms of action are important to improve the feasibility and scientific validity of the study results.

The combination of gemcitabine, oxaliplatin, and apatinib has been shown to enhance immune function, limit the proliferation and spread of tumor vascular cells, and attenuate the expression of sIL-2R and sICAM-1 in patients with gallbladder cancer. This is a safe and effective treatment for advanced gallbladder cancer, and it presents a new idea for clinical trials.

## Figures and Tables

**Figure 1:** Comparison of immune index levels.

**Figure 2:** Comparison of serum tumor markers.

**Figure 3:** Comparison of clinical efficacy.

**Figure 4:** Comparison of survival indicators.

**Figure 5:** Comparison of the incidence of adverse reactions.

**Table 1:** Comparison of immune index levels.

Group	Period	Observation group	Control group
		(*n* = 58)	(*n* = 58)
CD3+(%)	Before	47.92 ± 9.56	47.85 ± 9.58
	After	54.83 ± 11.97^*∗*^	62.97 ± 12.74^*∗*#^
CD4+(%)	Before	35.86 ± 6.98	35.87 ± 6.84
	After	40.15 ± 7.57^*∗*^	48.97 ± 8.12^*∗*#^
CD8+(%)	Before	25.12 ± 6.42	25.13 ± 6.48
	After	22.97 ± 5.14^*∗*^	16.89 ± 4.23^*∗*#^
CD4+/CD8+	Before	1.33 ± 0.29	1.35 ± 0.26
	After	1.58 ± 0.34^*∗*^	1.89 ± 0.52^*∗*#^
NK(%)	Before	16.89 ± 4.16	17.23 ± 4.39
	After	32.76 ± 6.98^*∗*^	37.89 ± 7.42^*∗*#^

**Table 2:** Comparison of serum tumor markers.

Group	Period	Observation group	Control group
		(*n* = 58)	(*n* = 58)
sIL-2R (IU/ml)	Before	763.02 ± 136.24	760.91 ± 135.43
	After	649.14 ± 115.68^*∗*^	528.32 ± 93.61^*∗*#^
sICAM-1 (*μ*g/l)	Before	513.21 ± 145.76	516.86 ± 148.97
	After	359.42 ± 112.64^*∗*^	218.54 ± 79.36^*∗*#^
VEGF (ng/ml)	Before	570.43 ± 106.94	573.54 ± 109.83
	After	403.21 ± 84.55^*∗*^	238.17 ± 69.31^*∗*#^
CEA (ng/ml)	Before	38.20 ± 10.93	38.41 ± 10.89
	After	23.01 ± 8.06^*∗*^	15.73 ± 4.88^*∗*#^

**Table 3:** Comparison of clinical efficacy.

Group	Observation group	Control group	*χ * ^2^ index	*P* index
	(*n* = 58)	(*n* = 58)		
CR	3(5.17)	8(13.79)	—	—
PR	11(18.97)	19(32.76)	—	—
SD	27(46.55)	22(37.93)	—	—
PD	17(29.31)	9(15.52)	—	—
RR	24.14%	46.55%	0.786	0.012
DCR	70.69%	84.48%	1.023	0.005

The article "Effects of Gemcitabine and Oxaliplatin Combined with Apatinib on Immune Function and Levels of SIL-2R and sicAM-1 in Patients with Gallbladder Cancer" was retracted in 2023. Reasons: signs of a paper mill; suspected computer-generated content; unreliable results or conclusions; concerns about the data.

**Table 4:** Comparison of survival indicators.

Group	Observation group	Control group	Statistical index	*P* index
	(*n* = 58)	(*n* = 58)		
Survival rate	39(67.24)	46(79.31)	0.201	0.014
Time (months)	8.15 ± 1.23	10.93 ± 1.26	4.303	0.021
PFs (months)	4.96 ± 1.15	5.43 ± 1.08	5.133	0.004
0s (months)	7.85 ± 1.04	9.53 ± 1.23	2.854	0.038

**Table 5:** Comparison of the incidence of adverse reactions.

Group	Observation group	Control group	*χ* ^2^ index	*P* index
	(*n* = 58)	(*n* = 58)		
Hypertension	11(18.97)	7(12.07)	5.402	0.340
Neutropenia	5(8.62)	1(1.72)	0.185	0.018
Proteinuria	7(12.07)	3(5.17)	0.892	0.006
Bone marrow depression	8(13.79)	3(5.17)	0.418	0.522
Hand-foot syndrome	6(10.34)	5(8.62)	0.322	0.023

## Data Availability

The data used to support the findings of this study are available from the corresponding author upon request.
